The article "The microRNA-325 inhibits hepatocellular carcinoma progression by targeting high mobility group box 1" was retracted in 2018. Reason: plagiarism.

# The microRNA-325 inhibits hepatocellular carcinoma progression by targeting high mobility group box 1

**DOI:** 10.1186/s13000-015-0323-z

**Published:** 2015-07-22

**Authors:** Huifen Li, Weihua Huang, Rongcheng Luo

**Affiliations:** Department of Chemotherapy, Zhongshan People’s Hospital, Zhongshan, Guangdong 528400 China; TCM-Integrated Hospital, Southern Medical University, Cancer Center, NO.13 Shiliugang Road, Haizhu District, Guangzhou, Guangdong 510315 China

**Keywords:** miR-325, HMGB1, Proliferation, Invasion, Hepatocarcinoma carcinoma

## Abstract

**Background:**

MicroRNAs (miRNAs) can serve as tumor suppressors and might provide an efficient strategy for annihilating tumor cells. Nevertheless, the potential role of miR-325 in hepatocellular carcinoma (HCC) is still unknown.

**Methods:**

Using RT-PCR, immunoblots invasion assays and bioinformatics strategies, we investigated the potential role of miR-325 in HCC.

**Results:**

We showed that miR-325 was decreased and HMGB1 was increased in 99 patients with hepatocellular carcinoma. MiR-325 inhibition promoted cell invasion and proliferation, while miR-325 upregulation inhibited cell invasion and proliferation by using transwell and CCK8 assays. We further showed that HMGB1 might be a direct target of miR-325 and is negatively regulated by miR-325. Down-regulation of miR-325 predicts poor prognosis for HCC patients.

**Conclusions:**

These findings implied that miR-325 regulates cell invasion and proliferation via targeting HMGB1 and may be a potential prognostic marker for HCC.

**Virtual slides:**

The virtual slide(s) for this article can be found here: http://www.diagnosticpathology.diagnomx.eu/vs/4655707031717989

## Background

Human hepatocellular carcinoma (HCC), one of the most common aggressive tumors worldwide has relatively high mortality rate among malignant tumors [1]. The overall 5-year survival rate for HCC is extremely low (18 %) [1]. Due to the lack of specific early symptoms or effective tumor biomarkers, most patients with HCC are diagnosed at the advanced stages. Even though there has been great improvement on traditional treatments, such as surgery supplemented with radiotherapy and chemotherapy, the prognosis of these patients is very poor. Thus, it is extremely necessary to identify novel and efficient biomarkers used in the diagnosis and as therapeutic targets for human HCC.

MicroRNAs (miRNA) are small noncoding RNA molecules that can function as a posttranscriptional factor for gene expression and determine cell fate by modulating multiple cellular pathways. The miRNAs may exert their functions by base-pairing with the 3’-untranslated region (3’-UTR) of target mRNAs [2]. Deregulated miRNAs are often indicators of cellular event that contribute to the onset of malignancy such as tumor [3]. A number of recent *in vitro* and *in vivo* studies have identified critical roles for miRNAs in the regulation of tumor cell invasion, metastasis and migration [4]. One potential reason that miRNAs are downregulated at many cancer cells is that they may target multiple oncogenic pathways and serve as tumor suppressors by inducing apoptosis. Downregulation of tumor suppressor miRNAs in various tumor tissues has been extensively reported [5–7]. Apoptosis is a complex process that proceeds through either intrinsic or extrinsic pathways [8]. The extrinsic pathway, which is triggered by death-ligand will culminate in effector caspase activation [9]. The intrinsic pathway centers on the mitochondria, which contain key apoptogenic factors such as cytochrome c, AIF, SMAC/DIABLO, Htra2/Omi [10]. Once activated, intricate interactions among BCL-2 family members can trigger the release of these factors and initiate effective apoptotic program [10].

High mobility group box 1 (HMGB1), the most important member of the high mobility group box protein family, is a nuclear protein with different functions in the cell; it has a role in cancer progression, angiogenesis, invasion, and metastasis development. For example, HMGB1 is a newly identified gene overexpressed in ovarian cancer and associated with poor pathologic features [11]. Furthermore, Zhang et al. reported that HMGB1 could facilitate lymphangiogenesis, while HMGB1 coculture with tumor associated macrophages may strengthen the pro-lymphangiogenic potential [12]. HMGB1 overexpression has a significant role in tumor progression (especially migration of tumor cells) and tumor ability to metastasize in colorectal cancers. Thus, it corroborates the idea that it might be an important prognostic factor [13]. Knockdown of HMGB1 inhibits growth and invasion of gastric cancer cells through the NF-κB pathway *in vitro* and *in vivo* [14].

In this study, we sought to investigate the potential role of miR-325 in patients with HCC. Furthermore, we verified that miR-325 could regulate cells invasion and proliferation of HCC by targeting HMGB1. Therefore, miR-325 may be a potential prognostic marker for HCC.

## Methods

### Clinical samples and statements

All the liver cancer tissues and correspondingly normal adjacent samples were collected from the 99 patients that had undergone routine surgery at TCM-Integrated Hospital, Southern Medical University from January 2010 to November 2013. Total tissues were stored at −80 °C until RNA extraction. Our study was approved by the Ethical Committee of TCM-Integrated Hospital, Southern Medical University and every patient has written informed consent, the study methodologies conformed to the standards set by the Declaration of Helsinki.

### Cell culture

The human hepatocellular carcinoma cell lines (SMMC-7721, Hep3B, HepG2, Huh7 and Bel7404) and normal liver cell (LO2) were purchased from the Institute of Biochemistry and Cell Biology of the Chinese Academy of Sciences (Shanghai, China). All cell lines were cultured in RPMI-1640 medium with 10 % fetal bovine serum (Invitrogen, Carlsbad, CA) and penicillin (200 U/ml) at 37 °C with 5 % CO_2_.

### Isolation of total RNA and Quantitative RT-PCR

RNA of all the tumor samples and corresponding adjacent tissues was extracted by using TRIzol (Invitrogen, Carlsbad, CA) and both miRNA and mRNA were reversely transcribed to cDNA. MiRNAs expression levels were detected by using the TaqMan stem-loop qRT-PCR method with a mirVana miRNA Detection Kit and gene-specific primers, and normalized to U6. Relative HMGB1 mRNA expression levels were examined by using SYBR Green quantitative real-time PCR (qRT-PCR). Genepharma synthesized the HMGB1 siRNA. And GAPDH was used for normalization. The following primers were used as follow.

- HMGB1: (forward) 5'-GCTCCATAGAGACAGCGCCGGG-3',
- (reverse) 5'-CCTCAGCGAGGCACAGAGTCGC-3'.
- siHMGB1: (sense) 5'-CCCGUUAUGAAAGAGAAAUTT-3',
- (antisense) 5'-AUUUCUCUUUCAUAACGGGTT-3'.

qRT-PCR assay was performed by using the ABI 7900 Fast Real-Time PCR system (ABI, CA, USA).

### Invasion assay

Invasion assays were conducted with BioCoat Matrigel (BD Biosciences, San Jose, CA) and invasion chambers (Millipore, Eschborn, Germany) with an 8-μm pore size according to the manufacturers’ instructions. The chamber were coated with 200 mg/ml BD Matrigel (BD Biosciences, Shanghai, China) and dried overnight. All the cell lines (5 × 10^5^) were incubated at 37 °C for 48 h before staining with crystal violet. A set of images was acquired by using NIS Elements image analysis software (Nikon, Tokyo, Japan). The values for invasion were obtained by averaging over three fields of view per well from a three replicate set of samples for each experimental condition [15].

### Cell-proliferation assay

Cells were seeded into 96-well plates (1.0 × 10^4^ cells per well). Cell viability was assessed by cell-counting kit-8 assay (Beyotime Institute of Biotechnology, Shanghai, China). The absorbance of each well was monitored by a spectrophotometer (Thermo, Shanghai, China) at 450 nm (A450). For each case, three independent experiments were performed.

### Apoptosis assay

Twenty-four hours after transfection with miR-325 mimics, NC, miR-325 inhibitor and inhibitor NC, the apoptosis in cultured cells was analyzed using annexin V labeling. An annexin V–APC labeled Apoptosis Detection Kit (Abcam, Shanghai, China) was used according to the manufacturer's protocol.

### Western blot

All the proteins were extracted from cultured cells, quantitated using a protein assay (bicinchoninic acid [BCA] method; Beyotime, Shanghai, China). Proteins were fractionated by sodium dodecyl sulfate polyacrylamide gel electrophoresis, transferred to polyvinylidene fluoride (PVDF) membrane, blocked in 5 % dry milk at room temperature for 1.5 h, and immunostained with primary anti-HMGB1 (1:1000, Sigma, Shanghai, China) and anti-GAPDH (1:5000, Kangchen, Shanghai, China). All results were visualized through a chemiluminescent detection system (Pierce ECL Substrate Western blot detection system, Thermo, Pittsburgh, PA) and then exposed in Molecular Imager ChemiDoc XRS System. The integrated density of the band was quantified by Image software (Bio-Rad, Hercules, CA).

### Transient transfection and Luciferase assay

Both oligonucleotides miR-325 mimics and hsa-miR-325 inhibitor (anti-miR-325) were purchased from GenePharma (Shanghai, China) along with NC (miR-control) and inhibitor NC (anti-miR-control). HepG2 and Huh7 cells were seeded into 6-well plates and transfected with 100 nM siRNA/HMGB1 and siRNA/control (GenePharma, Shanghai, China) using Lipofectamine 2000 (Invitrogen, NY, USA) at a final concentration of 100 nM. The transfection efficiency was monitored by using qRT-PCR. For the luciferase reporter assay, cells were cultured in 96 well plates and transfected with luciferase reporters (50 ng), and 50 nM of miR-control, miR-325 mimics or miR-325-mut. After 48 h, luciferase activity was measured using dual-luciferase reporter system (Promega, USA). The renilla activity was used as an internal control. Each transfection was performed in triplicate.

### Statistical methods

All values are expressed as mean ± SEM. Statistical analysis was performed using STAT10 and GraphPad Prism (version 5.01; GraphPad Software, Inc, La Jolla, CA) statistical software. The chi-squared test was used to test the significance of observed differences in the Table 1 data and the *t*-test was used for the other data analyses. The *p* values less than 0.05 were considered significant.

**Table 1:** The clinical characteristics relevance analysis of miR-325 and HMGB1 in patients with HCC

Characteristics	All Patients	miR-325 low Expression (≤ Median^a^)	miR-325 high Expression (> Median^a^)	*p* value	HMGB1 low Expression (< Median^b^)	HMGB1 high Expression (≥ Median^b^)	*p* value
NO.	99	51	48		49	50	
Age(years)				0.832			0.565
<60	43	21	22		23	20	
≥60	56	28	28		26	30	
Gender				0.713			0.442
Male	46	24	22		25	21	
Female	53	26	27		24	29	
Histology				0.523			0.718
AC	45	23	22		21	24	
SCC	54	28	26		27	27	
Tumor size				0.003*			0.001*
T1/T2	46	17	29		35	11	
T3/T4	53	37	16		18	35	
TNM stage				0.001*			0.000*
I-II	48	10	38		36	12	
III-IV	51	35	16		10	41	
Metastasis				0.000*			0.000*
Yes	33	27	6		4	29	
No	66	23	43		45	21	

^a^median = 0.5115

^b^median = 3.0011

*denotes *p* value < 0.05

AC: adenocarcinoma; SCC: squamous cell carcinoma; HCC: hepatocellular carcinoma

## Results

### The miR-325 is reduced and HMGB1 is elevated in HCC tissues

First, we detected the expression levels of miR-325 and HMGB1 in HCC specimens (*n* = 99) as compared with corresponding adjacent tissues (*n* = 99) by using qRT-PCR. Significantly, we discovered that lower miR-325 (*p* < 0.05; Fig. 1a) and higher HMGB1 (*p* < 0.05; Fig. 1a) mRNA levels were expressed in HCC tissues than those in adjacent tissues. All patients were divided into two groups using median RNA level of miR-325 (^a^median = 0.5115) and HMGB1 (^b^median = 3.0011) as threshold, respectively. We found that the expression of miR-325 was negatively correlated with HMGB1 expression (R = −0.4725; *p* = 0.0003) in cancer samples (Fig. 1b). The expression of miR-325 was highly associated with HCC tumor size, TNM stage and metastasis of patients (Table 1), which suggests that that miR-325 may play an important role in the pathogenesis of HCC.

**Fig. 1:** miR-325 is decreased and inversely relates to HMGB1 expression in HCC patients. **a** Box-plot analysis of miR-325 and HMGB1 levels in 99 HCC patient samples and corresponding adjacent tissues. T refers to tumor tissues and P refers to corresponding adjacent tissues. **b** A negative correlation was found between RNA expression of miR-325 and HMGB1 in tumor samples (*P* < 0.0001). **c** Kaplan–Meier overall and progression-free survival curves for liver cancer patients with high and low miR-325 expression. Liver cancer patients with low miR-325 expression had significantly shorter overall (*P* < 0.05) and progression-free (*P* < 0.05) survival than those with high miR-325 expression did. Data were shown as mean ± SEM of three independent experiments. * indicates *P* < 0.05

### Prognostic implications of miR-325 expression in HCC

To detect the prognostic implications of miR-325 expression in Overall Survival and Progression-free Survival of HCC, detailed clinical information of all 99 HCC patients in high miR-325 expression and low miR-325 expression groups was evaluated. Kaplan-Meier analysis demonstrated that HCC patients with lower miR-325 expression had significantly shorter Overall (*P* < 0.05, Fig. 1c) and Progression-free (*P* < 0.05, Fig. 1c) Survival than those with higher miR-325 expression. Moreover, the univariate analysis revealed that both the TNM stage (*P* = 0.019) and low miR-325 expression (*P* < 0.05) predicted poorer overall survival of HCC patients. Furthermore, the multivariate analyses identified clinical stage (*P* = 0.023) and miR-325 expression (*P* = 0.021) in HCC as independent prognostic factors for overall survival of HCC patients (Table 2).

**Table 2:** Univariate and multivariate analysis of overall survival in HCC patients (n = 99)

Variables	Univariate analysis			Multivariate analysis		
	HR	95 % CI	p value	HR	95 % CI	*p* value
Age	1.461	0.811-2.627	0.193	1.513	0.790-2.631	0.178
Gender	1.029	0.586-1.792	0.941	0.967	0.533-1.798	0.876
Histology	1.022	0.556-1.796	0.913	1.047	0.569-1.892	0.823
TNM Stage	1.934	1.123-3.454	0.019*	1.920	1.092-3.394	0.023*
miR-325 expression	1.731	1.000-3.128	<0.050*	1.952	1.101-3.476	0.021*

*:p<0.05 was considered significant

### miR-325 inhibits HCC cell invasion

Next, to clarify the role of miR-325 in HCC, we performed a transwell invasion assay in vitro. First, we analyzed miR-325 expression in five HCC cell lines (SMMC-7721, Hep3B, HepG2, Huh7 and Bel7404) as compared with a normal liver cell line (LO2) by using qRT-PCR assay. The assay showed that miR-325 level in those cancer cell lines was significantly downregulated compared with normal control (Fig. 2a). Among those cancer cells, HepG2 showed the lowest expression of miR-325 while miR-325 was highest in Huh7 (Fig. 2a). Based on this expression pattern, we chose the HepG2 and Huh7 liver cancer cells to explore the functions of miR-325 in HCC. The cell lines were transfected with NC (mimics negative control), miR-325 mimics, inhibitor NC and miR-325 inhibitor respectively. The efficiency of transfection was examined by using qRT-PCR assay (Fig. 2b). We found that up-regulation of miR-325 inhibited cell invasion (Fig. 2c). In addition, down-regulation of miR-325 expression promoted the invasive ability of HCC cell lines (Fig. 2c). These results suggested that the abnormal expression level of miR-325 may be capable of regulating HCC cell invasion.

**Fig. 2:** Aberrant expression of miR-325 regulates HCC cell lines invasion. **a** Expression of miR-325 was analyzed in five liver cancer cell lines (SMMC-7721, Hep3B, HepG2, Huh7 and Bel7404) and normal liver tissue (LO2). **b** The results of miR-325 expression in cell lines transfected with miR-325 mimics, miR-325 inhibitor, control for miR-mimics (NC) and control for miR-325 inhibitor (inhibitor NC) were validated by using qRT-PCR. **c** Transwell assay was performed according to the Material and Methods. HepG2 and Huh7 were treated with miR-325 mimics, miR-325 inhibitor, NC and inhibitor NC for 24 h. The representative images of invasive cells at the bottom of the membrane stained with crystal violet were visualized as shown. The quantifications of cell invasion were presented as percentage of cell numbers. Data are shown as mean ± SEM of three independent experiments. * indicates significant difference compared with control group (*P* < 0.05)

### Aberrant expression of miR-325 regulates cell proliferation in vitro

In order to detect the functional roles of miR-325, we further investigated the effect of miR-325 on proliferation by using CCK8 assay. The assay showed differences on proliferation after manipulation of miR-325 in both HepG2 and Huh7 cells at 12-h, 24-h, 48-h and 72-h (Fig. 3a). In both HepG2 and Huh7 cells, the proliferation was repressed in miR-325 mimics expressed cells, whereas downregulation of miR-325 expression had the reverse effect (Fig. 3a). In addition, we used flow cytometry analysis to examine whether miR-325 was involved in apoptosis. However, the assay showed that miR-325 did not affect apoptosis as compared with the control (Fig. 3b). These results indicated that aberrant expression of miR-325 could regulate cell proliferation but have no effect on apoptosis in HCC cell lines.

**Fig. 3:** miR-325 inhibits cell proliferation. **a** Absorbance at 490 nm was presented for HepG2 (left) and Huh7 (right), respectively. **b** Flow cytometry assay was used to analysis cell lines apoptosis. HepG2 (left) and Huh7 (right) * indicates P < 0.05

### HMGB1 was the direct targets of miR-325

Since miR-325 contributed to the development of HCC, we next set out to determine the potential mechanism in which miR-325 could affect cell proliferation and invasion in HCC cell lines. Based on the regulation pattern of miRNAs in human carcinoma, we explored the candidate genes which have been reported to be associated with cell invasion as well as regulated by microRNAs. We then predicated the potential target genes of miR-325 by using different bioinformatics analysis, microRNA.org (http://www.microrna.org/microrna/), miRDB (http://mirdb.org/miRDB/), and TargetScan (http://www.targetscan.org/) database. Finally, bioinformatic software indicated that 3'-UTR (untranslated region) of HMGB1 binds to miR-325 with the high score (mirSVR score: -1.1355). The predicted binding of miR-325 with HMGB1 3’UTR is illustrated in Fig. 4a (top panel). To further explore whether the suppression of HMGB1 expression induced by introducing miR-325 mimics was due to the binding of miR-325 to the 3'-UTR of HMGB1, we cloned the 3'-UTR fragment containing the predicted binding sites into pGL3 luciferase reporter vector (pGL3-HMGB1) according to the prediction. In the predicted target site, the 3ʹ-UTR fragment with mutant sequence was also cloned (pGL3-HMGB1-MUT) (Fig. 4a, top panel). The luciferase reporter assay showed remarkably reduced activity with miR-325 mimics and pGL3-HMGB1 vectors as compared with the control and all the mutant types (Fig. 4a, bottom panel). Moreover, to further confirm that miR-325 influenced HMGB1 expression, we performed qRT-PCR and western blot analyses. The results showed that in both mRNA and protein levels, up-regulation of miR-325 decreased HMGB1 expression; on the other hand, inhibition of miR-325 raised HMGB1 levels (Fig. 4b). These results suggested that miR-325 modulates HMGB1 expression by directly targeting its 3'-UTR.

**Fig. 4:** HMGB1 was the direct targets of miR-325. **a** The potential miR-325 seed region at the 3'-UTR of HMGB1 mRNA was predicted by using multiple bioinformatics analyses. HepG2 cells were co-transfected with miR-325 mimics (or NC) with pGL3-HMGB1 (or pGL3-HMGB1-mut) vector. Luciferase activity was normalized by the ratio of firefly and Renilla luciferase signals. **b** HMGB1 mRNA and protein expression levels in HepG2 (left) and Huh7 (right) cells transfected with NC, miR-325 mimics, inhibitor NC and miR-325 inhibitor were detected by using qRT-PCR and western-blotting. GAPDH was regarded as an internal control. Data are shown as mean ± SEM of three independent experiments. * indicates significant difference compared with control group (*P* < 0.05)

### Down-regulation of HMGB1 by siRNA partially reverses the promotion of cell invasion and proliferation induced by down-regulated miR-325

Furthermore, to explore whether the functional effect of miR-325 on HCC cell lines was dependent on HMGB1, we performed a rescue experiment. In the previous study, HMGB1 was increased in cells transfected with miR-325 inhibitor. So, we used RNA interference to silence the expression of HMGB1. *In vitro*, cell lines were co-transfected with miR-325 inhibitor and siRNA/HMGB1. The transfection cells with miR-325 inhibitor and the co-transfection cells with both miR-325 inhibitor and siRNA/control were regarded as the control groups. The western blot assay was used to examine the transfection efficiency (Fig. 5a). Furthermore, both the CCK8 assay and transwell invasion assay showed that down-regulation of HMGB1 partially attenuated the invasion and proliferation induced by miR-325 inhibition as shown in Fig. 5b and c, respectively. These results suggested that HMGB1 downregulation may potentially reverse the adverse effect induced by miR-325 inhibition.

**Fig. 5:** Down-regulation of HMGB1 by siRNA partially reverses the promotion of cell invasion and proliferation induced by miR-325 inhibition. **a** The transfection efficiency was validated by using western-blotting for both HepG2 and Huh7 cells transfected with miR-325 inhibitor and inhibitor + siRNA/HMGB1 (the co-transfection cells of miR-325 inhibitor and siRNA/HMGB1) and inhibitor + siRNA/control (co-transfected with miR-325 inhibitor and siRNA/control). GAPDH was used as a control. Averages of three independent experiments were shown in the histogram (right panel). **b** Absorbance at 490 nm was presented with Mean ± SEM. HepG2 (left) and Huh7 (right). **c** Transwell assay was performed as described in Material and Methods. Cells were treated with miR-325 inhibitor and inhibitor + siRNA/HMGB1 (the co-transfection cells of miR-325 inhibitor and siRNA/HMGB1) and inhibitor + siRNA/control (co-transfected with miR-325 inhibitor and siRNA/control) for 24 h. The representative images of invasive cells stained with crystal violet were shown at the bottom. * indicates *P* < 0.05

## Discussion

In this study, we have demonstrated that HCCs have a significantly different miR-325 expression profile when compared to normal hepatocellular cells. Accumulating evidence suggests that deregulation of miRNAs has been frequently observed in tumor tissues. These miRNAs have regulatory roles in the pathogenesis of cancer [16, 17]. Indeed, patients with liver cancer often exhibit tumor cell invasion and metastasis before diagnosis, which renders current treatments including surgery, radiotherapy, or chemotherapy ineffective. Therefore, studying the molecular basis of liver cancer is crucial for designing new therapeutic agents to improve the survival rate.

The miRNAs can bind target mRNAs at complementary sites in their 3'-untranslated regions (3'-UTRs), thereby suppressing the expression of the target gene at the posttranscriptional level. Through this mechanism, miRNAs regulate a wide range of biological processes [18]. For example, miR-545 suppresses cell proliferation by targeting Cyclin D1 and CDK4 [19]. The miRNAs can also predict the prognosis of patients with various cancers and may be a potential prognostic marker for cancers [20–22]. It was shown that the microRNA-125b inhibits the tumorigenic properties of HCC cells and may serve as a prognostic biomarker [23]. Up-regulation of microRNA-183-3p is a potent prognostic marker for lung adenocarcinoma of female non-smokers [24]. miR-10b expression was an independent prognostic factor in lung cancer patients [25]. Shiiba et al. showed that miR-325 might play a role in head and neck squamous cell carcinoma [26]. In addition, Tang et al. suggested that the miR-325 may potentially function as a prognostic marker for prostate cancer [27]. To date, very few reports have demonstrated the role of miR-325 and its association with tumor characteristics especially for HCC. In a microRNA expression profiling study, Wong et al. implied that miR-325 might be involved in HCC malignancy [28]. However, the exact or potential mechanisms have not been investigated. Here we showed that the expression of miR-325 was significantly decreased in HCC tissues (Fig. 1). Aberrant expression of miR-325 was related to the invasion and proliferation of HCC cell lines (HepG2 and Huh7) *in vitro*. Patients with low miR-325 expression had poorer survival than those with high miR-325 expression. Furthermore, we also found that miR-325 overexpression diminished but miR-325 knockdown increased HMGB1 expression level in HCC cell lines by directly binding to the 3'-UTR of HMGB1. Similarly, we tried to elucidate the reverse regulation of miR-325 and HMGB1 within HCC, but we are unsure whether miR-325 has other targets related to HCC proliferation and invasion. These results suggested that changes in the development of HCC should not be attributed to alternations of one or a small number of genes. As the limit on the number of HCC samples and cell types, more elaborate studies will be necessary for further exploration of the link between miR-325 and HMGB1 and potential roles of miR-325 in tumorigenesis.

HMGB1 is initially defined as chromatin-related protein with high acidic and basic amino acid content [29]. A recent study reported that HMGB1 modifies the interaction of DNA with transcription factors like p53 steroid hormone receptors by non-specifically binding to a smaller groove of DNA, and this is related to DNA repair, transcription, differentiation, extracellular signalization, and somatic recombination [30]. Evidence supporting the role of HMGB1 in cancer progression, angiogenesis, invasion, and metastasis development has been steadily accumulating [31]. Existing studies suggest that HMGB1 may have an important role in tumor progression beyond cancer development. The association of HMGB1 overexpression with lymph node metastasis, advanced stage in head-neck, esophagus squamous cell carcinoma, and cervix uteri has been demonstrated [32–34]. All their findings supported the view that HMGB1 may function as an oncogene. Here, we found that HMGB1 was overexpressed in HCC samples and associated with metastasis. Furthermore, we found that silencing HMGB1 by siRNA partially abolished the enhancement of cells invasion and proliferation induced by down-regulation of miR-325. These results implied that the functional effect of miR-325 on HCC was dependent on HMGB1.

An accurate prognosis is essential, particularly in malignant diseases, to provide advice to patients and guidance for assessment and treatment. Clinical evaluation and therapeutic decisions in HCC is complex because they depend on both the grade of cancer spread (tumor staging) and residual liver function (chronic liver disease stage). A majority of patients with HCC are diagnosed at a late stage, and only a small percentage fit resection or transplantation criteria. Although well-defined and generally accepted staging systems are available for almost all cancers, HCC is an exception, with many different staging systems globally introduced to accommodate each stratum of the disease [35–37]. Thus, an accurate predictor of prognosis and a sensible selection criterion that can be applied to patients with HCC, particularly with early stage HCC, for rational treatment decisions remains a challenging task. The miR-325 signature identified in this study significantly correlates with survival of patients with HCC with relatively small tumors who might be at an early stage of this disease. In contrast, the clinical HCC staging systems were unable to distinguish the outcome of these patients in this cohort. Our results suggest that the miR-325 signature may be a useful tool to classify patients with HCC assisting in their diagnosis and improving clinical outcome.

## Conclusions

In conclusion, we here provide evidence that reduced expression of miR-325 may contribute to cell proliferation and invasion in HCC by directly targeting HMGB1. Moreover, miR-325 was frequently downregulated in HCC and decrease in miR-325 was significantly correlated with poor prognosis of patients with HCC., therefore miR-325 might be utilized as a diagnostic marker in future.
